The article "Diagnosis, classification and grading of canine mammary tumours as a model to study human breast cancer: an Clinico-Cytohistopathological study with environmental factors influencing public health and medicine" was retracted in 2016. Reasons: plagiarism; compromised peer review; concerns about the authorship.

# Diagnosis, classification and grading of canine mammary tumours as a model to study human breast cancer: an Clinico-Cytohistopathological study with environmental factors influencing public health and medicine

**DOI:** 10.1186/1475-2867-13-79

**Published:** 2013-08-09

**Authors:** Radmehr Shafiee, Javad Javanbakht, Nahid Atyabi, Pegah Kheradmand, Danial Kheradmand, Alimohammad Bahrami, Hasti Daraei, Farshid Khadivar

**Affiliations:** 1 Faculty of Veterinary Medicine, Tehran University, Tehran, Iran; 2 Department of Pathology, Faculty of Veterinary Medicine, Tehran University, Tehran, Iran; 3 Semnan University of Medical Science, Faculty of Medicine, Semnan, Iran; 4 MD, Graduate Islamic Azad University of Mashhad, Faculty of Medicine, Mashhad, Iran; 5 MD, Graduate Paraveterinary Faculty of Ilam, University of Ilam, Ilam, Iran; 6 Department of Environmental Health Engineering, Alborz University of Medical Sciences, Karaj, Iran

**Keywords:** Grading of tumours, Cytohistopathology, Dog, Mammary glands, Tumour

## Abstract

**Background:**

The human “Elston and Ellis grading method” was utilized in dogs with mammary tumor to examine its relation to prognosis in this species, based on a 2-year follow-up period. Although cytopathology is widely used for early diagnosis of human neoplasms, it is not commonly performed in veterinary medicine. Our objectives in this study were to identify cytopathology criteria of malignancy for canine mammary tumors and the frequency of different types of mammary lesions and their relationship with histologic grade was investigated. Another aim of this study was to differentiate the simple and adenocarcinoma tumors from the complex or mixed tumor described by Elston and Ellis grading method.

**Methods:**

The study was performed in 15 pure or mixed-breed female dogs submitted to surgical resections of mammary tumours. The mammary tumours were excised by simple mastectomy or regional mastectomy, with or without the superficial inguinal lymph nodes. Female dogs were mainly terriers (9 dogs) or mixed (3 dogs), the 3 other animals were a German shepherd, Dachshund and Pekingese. Before surgical excision of the tumour, FNAC was performed using a 0.6 mm diameter needle attached to a 10 ml syringe held in a standard metal syringe holder. The cytological sample was smeared onto a glass slide and either air-dried for May-Grünwald-*stain,* or ethanol-fixed for Papanicolaou stain and masses were surgically removed, the tumours were grossly examined and tissue samples were fixed in 10%-buffered-formalin and embedded in paraffin. Sections 4 μm thick were obtained from each sample and H&E stained.

**Results:**

We obtained a correct cytohistological correlation in 14/15 cases (93.3%) when all cytopathological examinations were considered. Of the 15 cases examined, 2(13.3%) had well-differentiated (grade I), 6(40%) had moderately differentiated (grade II) and 7(46.7%) had poorly differentiated (grade III) tumours. Classification of all canine mammary gland lesions revealed 13(86.7%) malignant and 2(13.3%) benign tumors. The histological examination showed that the most common tumor types of mammary glands in bitches were: complex carcinoma, adenocarcinoma, malignant mixed tumour, benign mixed tumour, simple carcinoma– (5/15; 33.3%), (3/15; 20%), (3/15; 20%) and (2/15;13.3%), respectively. Simple carcinoma and *cystic hyperplasia* were less common - (1/15; 6.7%), and (1/15; 6.7%), respectively. Moreover, the most often tumors occur in inguinal mammary (60%) and abdominal (27%) glands.

**Conclusions:**

Our results demonstrate that, because of the similarity of the cytohistopathological findings in the human and canine mammary gland tumours, it is possible to use the same cytopathological criteria applied in human pathology for the diagnosis of canine mammary gland tumours. Furthemoer, routine use of this human grading method would help the clinician to make a more accurate prognosis in the interests of post-surgical management in dogs with mammary carcinomas. Furthermore, this research will allow a more discriminating classification of mammary tumors and probably has a bearing on cytohistopathology, epidemiology, pathogenesis and prognosis. The most often tumors occur in inguinal mammary (60%) and abdominal (27%) glands. This interesting regional difference may be due to a) the duration of the growth before the diagnosis; b) the age of the dogs; and c) high prevelance of unspayed animals. Moreover, the most common type of tumor was complex carcinoma – 33.3% (5 cases).

## Background

Mammary gland tumours are one of the most common neoplasms in female dogs [1]. These spontaneous tumors are very similar to those in humans, but the incidence rate among bitches is 3 times larger than in women [2], and there are some molecular and biological similarities between canine and human mammary tumours [1-4]. Malignant cases occur in approximately half of canine mammary tumours (CMTs) [5,6], with a 3-fold higher incidence when compared with breast tumours in human females.2 Similar to their human counterparts, these tumours occur almost exclusively in females, and only rarely in male dogs [2]. Generally, in canine malignant mammary tumours (CMMT), metastatic spread occurs via lymphatic vessels to the regional lymph nodes or haematogenously and the lungs are the most frequent site of distant metastases [7].

A number of new methods are therefore tested within tumor pathology to improve the diagnostic and prognostic accuracy. To make a diagnosis, a number of clinical and paraclinical tests are used because it is essential to find the most aggressive malignant tumors that need radical surgery and supplementary treatment as soon as possible. After excision, a hematoxylin-eosin stain is often used to provide a histopathological diagnosis, but even though this is performed by experienced pathologists, the disorderly structure of some mammary tumors may cause confusion and may lead to an erroneous diagnosis of malignancy [8-11].

Anamnesis and physical examination coupled with epidemiological findings have an important role in the diagnosis and prognosis. Radiographic screening, surgical biopsy or aspiration biopsy are beneficial tools for early diagnosis of tumours. Although the first attempt is to make a differential diagnosis with inflammation or hyperplasia these tools should be used to understand the biological behavior of the mass that also contribute to the prognosis [12].

Cytological examination has important benefits in clarifying some aspects in early diagnosis of mammary lesions. This procedure is commonly used in palpable lesions such as mammary glands, thyroid, lymph nodes and salivary glands. It also prevents the need for a surgical attempt and complications that might occur during surgery [13]. Fine needle aspiration cytology (FNAC) is a method largely used to obtain samples for cytological diagnosis in several organs. When applied to mammary gland lesions, the method shows good diagnostic accuracy. Moreover, it is a simple, rapid and low cost method, with minimal risk for the patient [11-13]. Paget (1854) [14] was the first to use samples of aspirated mammary tumours for microscopic examination. In veterinary medicine, the use of cytology as a diagnostic method is very recent and has been growing in the last 20 years [7].

Our objectives in this study were to identify cytopathology criteria of malignancy for canine mammary tumors and the frequency of different types of mammary lesions and their relationship with histologic grade was investigated. Another aim was to differentiate the simple tumor from the complex or mixed tumor described by Elston and Ellis grading method.

## Results

### Macroscopic details and findings

The macroscopic specifications of the multifarious mammary masses were summarized in the Figure 1 and Table 1. The preferential localisation of mammary neoplasms were the inguinal lobes (60% of cases), abdominal lobes (%27) and thoracic lobes (%13). Furthermore, 45% of the inguinal masses affected the cranio-inguinal lobe, %33 caudo-abdominal lobe and %22 cranio and caudo abdominal lobes, whereas thoracic masses were found in two cases and abdominal masses in four of cases. Eventually, % 67 of tumour masses were found in the left mammary lobes and %33 in the right mammary lobes. Eighty % of mammary tumours exhibited a small size, with weight inferior to 50 g but a relatively high proportion of these masses (20%) weighted more than 100 g, even reaching 110 g and 180 g (cases n° 13 and 17 respectively). The majority of the tumours showed a hard or an elastic consistency but some of them appeared fluctuant (cases n°3, 6 and 8). In the great majority of cases (93%), the aspect of the tumour on the cut surface was grayish-white and lobed. Some cystic structures or blood spot districts areas were also often found (in 40% and 20% of cases, respectively) (Figure 1).

**Figure 1:** The relative risk of neoplasms of the mammary gland in female dogs in individual age and tumor size categories.

**Table 1:** Cytological and histopathological analysis of pre-operative and sampled during surgery from the mammary neoplasms of the 15 females dogs together with signalment of bitches included in the this study

**The number of cases of mammary tumours in 15 female dogs**	**Tumour localisation**	**Cytological type**	**Cytological classification**	**Histopathological type**	**Histopathological classification**
1	Right cranio and caudo inguinal lobes / left caudo-inguinal lobe	carcinoma	Malignant	Complex carcinoma	Malignant
2	Left thoracic lobe	carcinoma	Malignant	Malignant mixed tumour	Malignant
3	Left cranio abdominal lobe	Benign secretory	Benign	Benign mixed tumour	Benign
4	Left cranio and caudo inguinal lobes	carcinoma	Malignant	Complex carcinoma	Malignant
5	Right cranio inguinal lobe	carcinoma	Malignant	Complex carcinoma	Malignant
6	Left caudo inguinal lobe	carcinoma	Malignant	Simple carcinoma	Malignant
7	Left cranio inguinal lobe	adenocarcinoma	Malignant	Malignant mixed tumour	Malignant
8	Left cranio and caudo inguinal lobe and right caudo-inguinal lobe	carcinoma	Malignant	Complex carcinoma	Malignant
9	Right caudo inguinal lobe	Benign secretory	Benign	Benign mixed tumour	Benign
10	Left cranio inguinal lobe	carcinoma	Malignant	Complex carcinoma	Malignant
11	Left cranio and caudo abdominal lobes	carcinoma	Malignant	Solid adenocarcinoma	Malignant
12	Right cranio inguinal lobe	hyperplasia	Benign	Cystic hyperplasia	Malignant
13	Left cranio inguinal lobe	carcinoma	Malignant	Malignant mixed tumour	Malignant
14	Right cranio-abdominal lobe	adenocarcinoma	Malignant	Papillary adenocarcinoma	Malignant
15	Left thoracic lobe	adenocarcinoma	Malignant	Solid adenocarcinoma	Malignant

### Cytology findings

All the tumor masses were divided into four cytologic groups: hyperplasia (one case), adenocarcinoma (2 cases), carcinoma (9cases), benign secretory (3 cases) (Figure 2).

**Figure 2:** Cytological analysis of pre-operative fine needle aspirates and histopathological analysis of mammary tumour masses sampled during surgery in the 15 females dogs.

In all cases with malign characteristics (malign (dogs n°2,4,5,6,8,10,11,12,13 and 15), and malign suspected masses(dogs n°1,7 and 14)), clusters of cells with anisocytosis, anisokaryosis and hyperchromasia were observed (Figure 3A).

In the other malignant tumours, some nuclear anomalies were identified such as double nucleus in 8 samples (53%) of malignant tumours (Figure 3B, 3C, 3E and 3F), giant nucleus in 8 samples (53%), mitotic figures in 7 samples (46%) and abnormal chromatin structures in 4 samples (26%). In 5 cases spindle shaped cells were associated with tumour cells (33%) (Figure 3E and 3G). In the 2 benign tumours (dog n°3 and 9), the mammary gland structure remained uniform (Figure 3H).

**Figure 3:** **Evaluation of accuracy of fine needle aspiration cytology for diagnosis of canine mammary tumours. A:** Fine-needle aspirate from a mammary carcinoma in adog. Variation in cell (anisocytosis) and nuclear. (anisokaryosis) size are present, May-Grunwald-Giemsa staining method, 1000X. **B:** Adenocarcinoma: Malignant mammary epithelial cells: Fine needle aspirate with hypercellular pleomorphic, large hyperchromatic naked cells with coarse and abundant chromatin granules and vacuolar changes, May-Grunwald-Giemsa staining method, 1000X. **C:** Malignant multinucleated mammary epithelial cell; nuclei exhibit nuclear criteria of malignancy; nuclei superimposed and in different focal planes. May-Grunwald-Giemsa staining method, 1000X. **D:** Cytological appearance of spindle shape cells, May-Grunwald-Giemsa staining method, 400X. **E:** Myoepithelial cells (spindle shape) with abundant chromatin granules (red arrows) in adenocarcinoma, May-Grunwald-Giemsa staining method, 1000X. **F** and **G:** This cluster of cells shows multinucleated cells containing several irregularly sized nucleiare found in some cases, May-Grunwald-Giemsa staining method, 1000X. **H:** Fine-needle aspiration biopsy. Benign mammary tumor epithelial cell cluster. Cytological appearance of uniform epithelial cells, May-Grunwald-Giemsa staining method, 400X.

### Histopathology findings

All the tumor samples were divided into six histopathologic groups: hyperplasia (one cases), adenocarcinoma (3 cases), complex carcinoma (5), simple carcinoma (1), benign mixed tumor (2 cases), and malignant mixed tumor (3cases) (Figure 4A), adenocarcinomas was further divided into papillary (one adenocarcinomas), and solid (two adenocarcinomas) types. According to their maximum diameter, the tumours were classified as T1 in 8/15 (53.3%), T2 in 3/15 (20%) and T3 in 4/15 (26.7%) dogs. The most frequently represented tumour type was complex carcinoma (5/15; 33.3%), followed by adenocarcinoma (3/15; 20%), malignant mixed tumor (3/15; 20%), benign mixed tumor (2/15;13.3% cases), simple carcinoma (1/15; 6.7%)and cystic hyperplasia (1/15; 6.7%), as presented in Table 1 (Figure 2).

The histological grades of the 15 cases were as follows: grade I, 2(13.3%); grade II, 6(40%); grade III, 7(46.7%) with high mitotic index. The relationship between tumour grading and histological type is presented in Table 2. Of the 15 dogs in which mammary examination was performed, 2 had well-differentiated grade I tumours (Cystic hyperplasia and benign mixed tumour), 6 had moderately differentiated grade II (1 papillary adenocarcinoma, 3 complex carcinoma, 1 benign mixed tumour and 1 malignant mixed tumor) and 7 had poorly differentiated grade III (1 solid adenocarcinoma, 1 papillary adenocarcinoma, 1 simple carcinoma, 2 complex carcinoma and 2 malignant mixed tumor) (Table 2).

**Figure 4:** **Histopathological evaluation of mammary gland tumours in dogs. A:** Solid adenocarcinoma; The presence of neoplastic, mitotic and inflammatory cells (H&E, X 200.), **B:** Cartilage tissue cells due to metaplasia in malignant mixed tumour H&E, X 400. **C**: Myoepithelial reaction included with spindle shape cells in carcinoma, H&E, X 400. **D** and **E:** A cystic tumour of adenocarcinoma showing local invasion of interlobular connective tissue and note the high mitotic index and also different mitotic figures (H&E, (H&E, × 400 and 200). **F:** Papillary adenocarcinoma proliferating neoplastic epithelial cells in the form of papillary projections and presence of mitotic figures. H&E, 200×, **G and H:** Beinign mixed mammay tumour. Tumour tissue showing epithelial and myoepithelial components, 400×, **I:** The presence of neoplastics emboli within the dermal lympathic vessels, which was occasionally observed with some of the most aggressive adenocarcinoma, leads to blockage of the superficial dermal lymphatic drainage (H&E, X 200), **J:** Cholesterol cleft in malignant mixed tumour, (H&E, X 400). **K:** Cells exhibit variable numbers of mitoses are found; or, the second population of cells may have oval to fusiform vesicular nuclei with an extensive amount of eosinophilic cytoplasm and distinct cells margins (H&E, X 400) **L:** Haemorrhage foci and the central necrotic areas are interpreted as an indication that the neoplastic cells are growing faster and that there is therefore a higher risk of progression to invasive carcinoma (H&E, X 400).

**Table 2:** Relationship between histological grading and tumour type together with number and percentage of cases in 15 dogs with mammary tumour

**Histological type**	**Grade I**	**Grade II**	**Grade III**	**Total**
Cystic hyperplasia	1(6.7%)	_	_	1(6.7%)
Solid adenocarcinoma	_	_	1(6.7%)	1(6.7%)
Papillary adenocarcinoma	_	1(6.7%)	1(6.7%)	2(13.3%)
Simple carcinoma	_	_	1(6.7%)	1(6.7%)
Complex carcinoma	_	3(20%)	2(13.3%)	5(33.3%)
Benign mixed tumour	1(6.7%)	1(6.7%)	_	2(13.3%)
Malignant mixed tumor	_	1(6.7%)	2(13.3%)	3(20%)
Total	2(13.3%)	6(40%)	7(46.7%)	15(100%)

Of the 15 canine mammary cancers (CMTs) included, 13 of the 15 cases exhibited a range of morphologies, a highly pleomorphic cell population and polygonal were a prominent feature of all neoplasms, accounting for greater than 86.7%of the tumour cell population in most cases. Also, in the group of CMTs, 46.7% (7/15) of cases were composed of highly cellular areas with a homogeneous population of spindle cells (Figure 4B, 4C and 4D). On the other hand, a high mitotic rate (More than three mitotic figures per high-power field (400×) was identified in 73.37% (11/15cases), with atypical mitoses conspicuous in all tumours (Figure 3E and 4E). In addition, 11 of the 15 (73.37%) CMTs cases showed necrotic foci and10 of the 15 (66. 7%) CMTs cases showed infiltrates of various numbers inflammatory foci primarily consisting of lymphocytes, plasma cells, and neutrophils cells (Figure 4G).

Furthermore, in the group of CMTs, 66.7% (10/15) of cases exhibited haemorrhage localized in the different regions of the tumor tissue (Figure 4L). Most CMTs this study increased mitotic activity, cellularity, nuclear pleomorphism and the presence of lesional necrosis are ominous features and suggest an increased risk of local recurrence (Figure 4I). According to local invasiveness, 33.3% of the tumours (5 out of 15) were found (Figure 3K and 4J). In addition, the neoplastic cells within the blood vessels were observed as well (Figure 4I). Moreover, 7 of the 15(46.7%) CMTs cases revealed that these tissue sections were comprised of cancerous epithelial cells characterized by hyperchromasia, enlarged nuclei, prominent nucleoli of mammary gland. Also, 4 of the 15(26.7%) CMTs cases exhibited cholesterol clefts in the lumina of the ducts (Figure 4J).

## Discussion

Clinical and cytopathological similarities between canine mammary tumours and human breast cancer have been described in recent decades [7].

Considering the breed distribution, cross breeds, terrier, mixed, German shepherd, Dachshund and Pekingese were predominant, which is similar as in other studies [15-17]. The age at diagnosis ranged from 6 to 14 years, with a median of 10 years. This interval of risk age is in agreement with other studies [17-20].

Mammary tumors are the most common neoplasms in female dogs1. Malignant tumors may carry a poor prognosis and necessitate surgery. Few data are available on the value of cytologic examination as a diagnostic or prognostic tool for mammary tumors in dogs. FNAC is considered a fast, accurate and cost-effective method for the diagnosis of human mammary tumours [8-11]. However, the evaluation of its accuracy is poorly reported in veterinary medicine. There is a difference concerning the frequency of lesions diagnosed in human versus the canine mammary gland. We performed a validity study to further characterize sensitivity and specificity values, as well as the accuracy of FNAC in the diagnosis of CMTs.

In our study, we found 93.3% cytological and histological diagnostic agreement. In previously reported studies of the canine mammary lesions, the agreement between the cytological and histological diagnosis ranged from 25% to 47% [5,21-23]. These results are low when compared with results of studies of human breast lesions published by Choi et al. [24] and Ciatto et al. [25]. They described high levels of agreement between cytological and histological diagnoses, ranging from 64.8% to 74.1%. In addition, when the authors excluded the inconclusive cases, their level of agreement increased to 93.1 and 96.7%, respectively. The results were at variance with findings of Simeonov and Stoikov [26], who reported 84.6% of correlation between cytological and histological diagnoses of mammary tumours.

In some studies, the fine needle aspiration cytology specimens contained many individual bizarre, multi-nucleated, and/or giant cells having hyperchromatic pleomorphic nuclei, prominent nucleoli, and relatively abundant cytoplasm, admixed with numerous mitotic figures in a hemorrhagic or inflammatory background in human. A small amount of sheet-like or three-dimensional clusters of malignant cells coexisted [20,22].

Histopathologic examination is considered the gold standard for the diagnosis of CMTs. The histological analysis of CMTs usually includes a spindle cell component. However, according to Allen et al. 1986, the presence of spindle cells in cytological samples of breast neoplasms is not restricted to mixed tumours, as these cells may be observed in other breast lesions, including myofibroblastomas, fibromatoses and even spindle cell carcinomas [27]. Despite the similar cytological and histological features between canine and human mixed tumours of mammary gland, in canines, these tumours are very common, while in humans they are very rare. Most of the canine mammary tumours are benign or malign mixed tumours that are composed with epithelial and myoepithelial proliferations with generally cartilage, bone and squamous metaplasia [28]. Allen et al. 1986 reported that the existence of spindle shaped cells within cytological aspirates should not be limited to mixed tumours as these cells might also exist in other mammary lesions such as myofibroblastoma . Haziroglu et al., 2010, present spindle shaped cells reported in one case of malignant mixed tumour and in one case of complex carcinoma [29]. In the present study, spindle shaped cells were encountered in two cases of malignant mixed tumour, in two cases of complex carcinoma and in one cases of solid adenocarcinoma, agreeing in this way with the previous reports.

Histopathological examination of the biopsy specimens was established as the most reliable diagnostic approach and revealed the characteristics of the tumour in many terms, which included pleomorphism, mitotic index, differentiation level, presence of necrosis, and the stromal invasion (the infiltration with neoplastic cells of the blood and lymph vessels and the cutaneous and soft tissue and the sur-gical margins). This data have been accepted as a golden standard in diagnosis due to its great importance in terms of the biological behaviour and the prognostic outcome of the neoplasia [30].

According to some authors, [31-34] tumors might have the potential to feed themselves via alternative pathways by vascular channels covered by deregulated neoplastic cells.

The presence of neoplastic emboli within the dermal lymphatic vessels, which was occasionally observed with some of the most aggressive CMTs, leads to blockage of the superficial dermal lymphatic drainage. The outcome is a clinical presentation that resembles an inflammatory process (inflammatory mammary cancer), which has a poor prognosis and a rapid, fatal clinical course, since all the available treatments are usually palliative [35-37].

The central necrotic areas are interpreted as an indication that the neoplastic cells are growing faster and that there is therefore a higher risk of progression to invasive carcinoma [38,39].

Histopathological diagnosis of CMTs is crucial in prediction of tumour behaviour after surgical excision. Moreover, histopathologic typing of the tumour is also important in establishing a post-operative chemotherapy plan to increase the survival time following the surgery since several protocols have been used with success in dogs [40]. Various classification systems [41-43] have been developed to estimate the prognosis of the disease.

Several studies revealed that half (42.0-55.0%) of the surgically removed mammary tumors in bitches were malignant 7. Meuten reported that about 20.0-40.0% of bitches with mammary tumors developed malignant kinds. 49 Although Simeonov and Stoikov reported that only 19.0% benign and 81.0% mammary tumors were malignant [26]. Moreover, Tavasoly et al., 2013 reported that all samples (n = 37) were malignant. In the present study only 13.3% benign and 86.7% mammary tumors were malignant [44]. Tavasoly et al., 2013 reported, 86.5% (n = 32), and 13.5% (n = 5) of mammary tumors were carcinomas and sarcomas, respectively. The most frequently represented tumor type was simple carcinoma 56.8% (n = 21), followed by complex carcinoma 13.5% (n = 5), sarcoma 13.5% (n = 5), carcinoma arising from benign tumor 10.8% (n = 4) and special type of carcinoma 5.4% (n = 2).

Rezaie et al. found that 70.6% of bitches had tubulopapillary carcinoma, 23.5%- solid carcinoma, and 5.9% - cribriform carcinoma [45] . Ežerskytė et al. indicated that the most common tumor types of mammary glands in bitches were simple carcinoma, complex carcinoma and carcinosarcoma 46.0%, 27.0% and 13.0%, respectively [46].

In the present study, the most frequently represented neoplasm type was complex carcinoma (5/15; 33.3%), followed by adenocarcinoma (3/15; 20%), malignant mixed tumor (3/15; 20%), simple carcinoma (1/15; 6.7%)and cystic hyperplasia (1/15; 6.7%).

However, in spite of this high percentage of malignant mammary tumors, according to WHO classification, the vast majority of malignant tumors were well differentiated adenocarcinomas, mostly complex and tubulopapillary, whereas special types of carcinomas and sarcomas were rare, which is similar as in other studies [16,17,47-49].

The measurement of only one of the parameters (variations of nucleus dimensions, giant nucleus formation, nucleus / cytoplasm distortion and rate, nuclear pleomorphism, changes in chromatin structures (altered dimensions, irregular chromatin shapes in nucleus, clearing of the parachromatin areas), variation in nucleolus number, abnormal nucleolus shape and presence of macronucleolus, mitotic count) associated with histological grade is unlikely to provide powerful prognostic information [50-52]. Complete histological grading is therefore preferable to nuclear grading for accurate prognosis. In the present study the main criteria retained to determine malignancy were tubule formation, the nucleus pleomorphism and dimension and a significant variation in the mitotic rates.

Most grading systems of mammary carcinomas in dogs are a modification of the numeric method of Elston and Ellis.

In the present study, a correlation between histological type and grade was evident. Carcinomas with a comparatively favourable prognosis, such as Complex carcinomas [30,53], were usually of grade II or III. On the other hand, simple carcinoma (the most malignant type) was usually grade III. Similar observations were reported in human patients by Elston and Ellis [51].

Because of the diversity of histological typing criteria, grading methods and endpoints used in different studies on the prognostic value of histological grading in canine mammary cancer, the results of such studies are difficult to compare [5,42,53]. In the only study 58 similar to ours(Due to the high percentage of tumor growth in the grade III), 50% of dogs with grade I mammary tumours, 64% with grade II, and 79% with grade III died within 2 years of surgical treatment. These results differed from our findings, possibly due to the use of a less refined grading method and the inclusion of sarcomas, which have the least favorable prognosis of all mammary tumours [50,54].

## Conclusions

Our results demonstrate that, because of the similarity of the cytological findings in human and canine mammary gland tumours, it is possible to use the same cytological criteria applied in human pathology for the diagnosis of canine mammary gland tumours. This study is hoped to open the way up for further cytopathology studies.

This study demonstrated that the Elston and Ellis method of histological grading in canine mammary tumor is a reliable prognostic factor. That is correlated with histopathological classification. Histological grading of canine mammary carcinomas by the Elston and Ellis method was significantly related to prognosis, especially in cases of simple carcinoma. Its routine use should be helpful in indicating appropriate post-surgical treatment.

The estimation of the proliferative activity of tumours by well standardized mitotic counting techniques should have a central position in histopathology research and practice.

Tumors of the mammary glands were most common in 6 – 14 year old bitches.

The most often tumors occur in inguinal mammary (60%) and abdominal (27%) glands. This interesting regional difference may be due to a) the duration of the growth before the diagnosis; b) the age of the dogs; and c) high prevelance of unspayed animals.

The most common type of tumor was complex carcinoma – 33.3% (5 cases).

## Materials and methods

### Animals characteristics

The study was performed in 15 pure or mixed-breed female dogs submitted to surgical resections of ‘mammary tumours’ in the Veterinary School Hospital of Tehran University Faculty with the complaints of mass existence in different mammary lobes. The animals, aged 6–14 years (mean ± SD = 10.5 ± 1.8), showed with or without clinical or radiological evidence of distant metastasis. Female dogs were mainly terriers (9 dogs) or mixed (3 dogs), the 3 other animals were a German shepherd, Dachshund and Pekingese. They were selected from cases treated surgically between July 2011 and February 2013. The mammary tumours were excised by simple mastectomy or regional mastectomy [50], with or without the superficial inguinal lymph nodes.

### Cytological evaluation

Before surgical excision of the tumour, Fine needle aspiration cytology (FNAC) was performed using a 0.6 mm diameter needle attached to a 10 ml syringe held in a standard metal syringe holder. The cytological sample was smeared onto a glass slide and either air-dried for May-Grünwald-stain, or ethanol-fixed for Papanicolaou stain. Subsequently, dogs were induced with propofol (4 mg/kg, IV, Propofol, Abbott) and anaesthetized with isoflurane (2-3%, Isoflurane, Adeka) and masses were surgically removed, the tumours were grossly examined and tissue samples were fixed in 10%-buffered-formalin and embedded in paraffin. Sections 4 μm thick were obtained from each sample and H&E stained. The cytopathological criteria adopted were those proposed by Bibbo [55] and for histopathological analysis of tumors it was used the Veterinary [30] and Human [56] classification. We considered the histopathological diagnosis as the ‘gold standard.

### Clinical and histopathological evaluation

Tumour size: Mammary neoplasms were classified by size according to the World Health Organization Clinical Staging System TNM 19, as T1 (<3 cm maximum diameter), T2 (3–5 cm maximum diameter) and T3 (>5 cm maximum diameter). In cases of multiple tumours, the largest one was used as the basis for classification.

Tumour type: Representative sections of each tumour (from the central core to periphery) and the excised lymph nodes were fixed in 10% buffered formalin, processed by routine methods, embedded in paraffin wax, sectioned at 5 μm and stained with haematoxylin and eosin (HE). Histopathological findings were recorded and used to classify the tumours according to the criteria of a recently validated system [30]. In cases with multiple tumours, the most malignant one as defined by Misdorp [50] was recorded.

Tumour grade: Histological grading was performed on HE-stained sections. According to the Elston and Ellis method [51], the grade for each case was derived from an assessment of (1) tubule formation, (2) nuclear pleomorphism, and (3) mitotic counts, each feature being scored 1 to 3 points. The scores were then added to obtain the tumour grade, as follows: 3–5 points, well-differentiated (grade I); 6–7 points, moderately differentiated (grade II); 8–9 points, poorly differentiated (grade III). Grading was carried out by one veterinary pathologist and, without prior knowledge of the results, confirmed by a second pathologist.

### Classification of tumours

The final diagnosis was classified in the protocol according to the following five categories: (1) benign, (2) suspicious-probably benign, (3) suspicious-probably malignant, (4) malignant and (5) insufficient/inadequate material for the diagnosis. However, to establish a comprehensive histological correlation, the two categories of suspicious cases were classified in a generic group entitled ‘suspicious-not otherwise specified.

## Abbreviations

CMTs: Canine mammary tumours; CMMT: Canine malignant mammary tumours; FNAC: Fine needle aspiration cytology; HE: Haematoxylin and eosin.

## Competing interests

The authors declare that they have no competing interests.

## Authors’ contributions

NA and RSH participated in the histopathological evaluation, performed the literature review, acquired photomicrographs and drafted the manuscript and gave the final histopathological diagnosis and designed and carried out all the experiments. JJ is the principal investigator of the laboratory in which the research was performed and contributed to the interpretation of the data and writing of the manuscript. PKH, DKH, AMB, HD and FKH edited the manuscript and made required changes and wrote the manuscript. All authors have read and approved the final manuscript.
